RETRACTED

# The specific MYB binding sites bound by *Ta*MYB in the *GAPCp2/3* promoters are involved in the drought stress response in wheat

**DOI:** 10.1186/s12870-019-1948-y

**Published:** 2019-08-19

**Authors:** Lin Zhang, Zhiqiang Song, Fangfang Li, Xixi Li, Haikun Ji, Shushen Yang

**Affiliations:** College of Life Sciences, Northwest A&F University, Yangling, 712100 Shaanxi China

**Keywords:** Drought tolerance, *Triticum aestivum*, *TaGAPCp* promoter, TaMYB

## Abstract

**Background:**

Drought stress is one of the major abiotic stresses that affects plant growth and productivity. The *GAPCp* genes play important roles in drought stress tolerance in multiple species. The aim of this experiment was to identify the core cis-regulatory elements that may respond to drought stress in the *GAPCp2* and *GAPCp3* promoter sequences.

**Results:**

In this study, the promoters of *GAPCp2* and *GAPCp3* were cloned. The promoter activities were significantly improved under abiotic stress via regulation of Rluc reporter gene expression, while promoter sequence analysis indicated that these fragments were not almost identical. In transgenic Arabidopsis with the expression of the GUS reporter gene under the control of one of these promoters, the activities of GUS were strong in almost all tissues except the seeds, and the activities were induced after abiotic stress. The yeast one-hybrid system and EMSA demonstrated that TaMYB bound *TaGAPCp2*P*/3*P. By analyzing different 5′ deletion mutants of these promoters, it was determined that *TaGAPCp2*P (− 1312~ − 528) and *TaGAPCp3*P (− 2049~ − 610), including the MYB binding site, contained enhancer elements that increased gene expression levels under drought stress. We used an effector and a reporter to co-transform tobacco and found that TaMYB interacted with the specific MYB binding sites of *TaGAPCp2*P (− 1197~ − 635) and *TaGAPCp3*P (− 1456~ − 1144 and − 718~ − 610) in plant cells. Then, the Y1H system and EMSA assay demonstrated that these MYB binding sites in *TaGAPCp2*P (− 1135 and − 985) and *TaGAPCp3*P (− 1414 and − 665) were the target cis-elements of TaMYB. The deletion of the specific MYB binding sites in the promoter fragments significantly restrained the drought response, and these results confirmed that these MYB binding sites (AACTAAA/C) play vital roles in improving the transcription levels under drought stress. The results of qRT-PCR in wheat protoplasts transiently overexpressing *TaMYB* indicated that the expression of *TaGAPCp2/3* induced by abiotic stress was upregulated by TaMYB.

**Conclusion:**

The MYB binding sites (AACTAAA/C) in *TaGAPCp2*P/*3*P were identified as the key cis-elements for responding to drought stress and were bound by the transcription factor TaMYB.

RETRACTED

**Electronic supplementary material:**

The online version of this article (10.1186/s12870-019-1948-y) contains supplementary material, which is available to authorized users.

## Background

Glyceraldehyde-3-phosphate dehydrogenase, the key enzyme responsible for the sixth step of glycolysis, is widely present in various biological cells [1]. The enzyme is encoded by the *GAPDH* gene and has important functions in cells [2, 3]. In plants, GAPDH is often divided into phosphorylated and nonphosphorylated forms. Phosphorylated GAPDH can be divided into GAPA/B, GAPC and GAPCp according to its distribution in cells, in which GAPCp is present in nongreen plastids. Studies have shown that AtGAPCp may play an important role in Arabidopsis ABA signaling pathways [4]. The lack of *GAPCp* in plants could disrupt the synthesis of major metabolites such as carbon and nitrogen metabolism, glycine and glutamine [5]. Mutations in the *GAPCp* gene cause metabolic abnormalities in the triose phosphate transporter (TPT) [6]. One of the important functions of GAPCp is to provide 3-phosphoglycerate (3-PGA) for anabolic pathways in heterotrophic cytoplasts [7]. These findings show that stress-inducible GAPCp may play a key role in the abiotic-stress response and signaling pathways. We have identified five GAPCp cDNAs from wheat, and their expression is induced under drought stress [8]. However, the complete regulatory mechanism governing *GAPCp* expression under drought stress is far from known.

Since gene expression patterns are regulated by promoters, it is very important to identify the cis-acting elements in promoters [9]. The promoter is a DNA sequence upstream of the 5′-flanking region of the structural gene and is capable of specifically recognizing and binding RNA polymerase, which regulates the expression of downstream genes by binding to specific recognition sites of transcription factors [10]. Identification of cis-acting elements bound by specific transcription factors can reveal transcriptional regulatory mechanisms and gene expression patterns involved in environmental adaptation processes [11]. Studies have shown that the response of Arabidopsis HSP26 promoter to high temperature and abiotic stress can be satisfactorily determined by detecting the expression intensity of the GUS reporter gene after deletion of some promoter elements [12]. The repeated 5′-CACGTG-3′ sequence in the AtNCED3 gene promoter of Arabidopsis was confirmed to be an important cis-acting element of this gene in response to drought stress [13]. Recently, drought-related regulatory factors have been identified in wheat including TaRZF38/70/59/74, PIMP1 (MYB transcription factor), TaERA1/ERF3, TaSnRK2.4/2.8, TaWRKY2/9 and TaNAC2a [14–18]. Among them, the MYB proteins are a large family of transcription factors that have different functions in growth and response to environmental stress [19–21].

RETRACTED

MYB plays a vital role in the regulation of auxin-regulated genes by binding to its response elements [22]. AtMYB also plays an important role in drought and salt tolerance in Arabidopsis [23, 24]. In rice, the expression of *OsMYB2* is induced by cold, drought and salt stress [25]. GbMYB5 increases the response of cotton to drought stress [26]. In wheat, several *MYB* genes involved in a variety of drought responses have been identified [27], and transgenic Arabidopsis plants overexpressing *TaMYB* have increased resistance to drought compared to wild type [28].

In this report we cloned and analyzed the promoter regions of the *TaGAPCp2* and *TaGAPCp3* genes. In transgenic Arabidopsis, the activity of GUS driven by the *TaGAPCp2* and *TaGAPCp3* promoters was markedly induced under drought stress. Yeast one-hybrid library screening identified one interacting transcription factor, and the interactions between *TaGAPCp2*P*/3*P and TaMYB were further confirmed by yeast cotransformation and electrophoretic mobility shift assay (EMSA). By analyzing the sequences and a series of deletion mutants, we identified two MYB binding motifs in the *TaGAPCp2* and *TaGAPCp3* promoters, which are the key cis-acting elements for responding to drought stress.

## Results

### Cloning and sequence bioinformatics analysis of *TaGAPCp*2P/3P

The 1822 bp of *TaGAPCp2* 5’regulatory region and 2049 bp of *TaGAPCp3* 5’regulatory region were obtained by PCR and cloned into the PGEM-T Easy vector for sequencing. We searched for putative cis-acting elements in the promoter regions of these two genes using the databases Plant Cis-acting Elements (http://www.bioinformatics.psb.ugent.be/webtools/plantcare/html/) and Plant cis-acting regulatory DNA elements (PLACE; http://www.dna.affrc.go.jp/PLACE/) [29]. A number of regulatory elements responsive to drought and ABA were recognized in both gene’s promoter region, including ABA-responsive elements (ABREs), dehydration-responsive elements (DREs), W-box elements, and MYB and MYC binding sequences. In addition, gibberellin responsive elements (GAREs) were also identified (Fig. 1, Additional file 1; Figure S1).

**Fig. 1:** Location of putative cis-elements in *TaGAPCp2* and *TaGAPCp3* promoters. Transcriptional start site (+ 1) is shown in black arrowhead

### Activity detection of *TaGAPCp2*P*/3*P via agrobacterium-mediated transient expression analysis

The promoter regions were fused into the GUS reporter vector to detect their activities in tobacco leaves. Histochemical assays were performed and the results are shown in Fig. 2a, which revealed GUS activity in transgenic tobacco leaves. All tobacco leaves were stained blue color except for the wild-type leaves, which demonstrated that *TaGAPCp2*P*/3*P could drive the expression of the GUS reporter gene in tobacco leaves. The dual luciferase reporter vector is more accurate and reliable than the mono-luciferase reporter for testing promoter activity. The relative expression of Rluc from the *TaGAPCp2*P*/3*P constructs was significantly increased under water stress compared to the control when normalized by Fluc expression (Fig. 2b, c).

RETRACTED

**Fig. 2:** Analysis of *TaGAPCp2* and *TaGAPCp3* promoters activity under abiotic stresses. **a** GUS staining of *TaGAPCp2* and *TaGAPCp3* promoters in transiently transformed tobacco leaves. P: positive control (CaMV 35S promoter); WT: wild type. **b** Analysis of RLUC activity for *TaGAPCp2* and *TaGAPCp3* promoters in transiently transformed tobacco leaves in response to stress. **c** Analysis of RLUC activity for *TaGAPCp3* promoter in transiently transformed tobacco leaves in response to stress. The indicated values are the average of three independent experiments. The standard deviation (SD) is indicated at each point. Significant differences between treated and untreated (control) conditions were assessed with one-sided paired t-tests (*, *P* < 0.05; **, *P* < 0.01)

### Construction of promoter-reporter plasmids and Arabidopsis transformation

The expressions of hygromycin and the promoters were detected in Arabidopsis transformed with 1301-TaGAPCp2P/3P, but no expression was observed in wild type (Additional file 2: Figure S2). These results confirmed the transgenes were expressed following transformation.

Histochemical staining of transgenic Arabidopsis plants where GUS expression was driven by *TaGAPCp2*P/*3*P yielded a whole-plant perspective of promoter activity (Fig. 3). In 15-day-old Arabidopsis plants, strong GUS expression was present throughout the entire plant. GUS expression was much higher in the roots and leaves than in other parts of the heading stage plant. In the siliques, GUS expression was present in the pods but not in the seeds inside the pods. In the two-week-old transgenic Arabidopsis plants, the GUS activities of *TaGAPCp2*P*/3*P were all observably induced after abiotic treatments with for 24 h (Fig. 4). For *TaGAPCp2*P*/3*P, the GUS activities increased 1.8-fold and 2.1-fold after PEG treatment. After H_2_O_2_ treatment, the GUS activities of *TaGAPCp2*P*/3*P were induced to the 2.9-fold and 2.7-fold and after ABA treatment the GUS activities of *TaGAPCp2*P*/3*P were induced to the 2.4-fold and 1.7-fold. These results demonstrated that *TaGAPCp2*P*/3*P may have some meaningful drought-related cis-elements.

RETRACTED

**Fig. 3:** Histochemical staining of transgenic Arabidopsis *TaGAPCp2*P and *TaGAPCp3*P. **a** 15-day old plant; **b** Heading stage plant (5–6 weeks); **c** silique

**Fig. 4:** GUS enzymatic activity quantification of transgenic Arabidopsis 24-h after abiotic stresses. **a** Expression of the GUS gene driven by *TaGAPCp2* promoter. **b** Expression of the GUS gene driven by *TaGAPCp3* promoter. The indicated values are the average of three independent experiments. The standard deviation (SD) is indicated at each point. Significant differences between treated and untreated (control) conditions were assessed with one-sided paired t-tests (*, *P* < 0.05; **, *P* < 0.01)

### *TaGAPCp2/3* could positively respond to drought stress in transgenic Arabidopsis plants

To determine if *TaGAPCp2/3* genes were important for drought stress tolerance, we evaluated drought stress responses in transgenic Arabidopsis plants overexpressing *TaGAPCp2/3* gene under control of the strong 35S promoter. Three-week-old seedlings of transgenic and WT plants were subjected to water stress for 25 days. We found that, WT plants were more sensitive to drought stress than transgenic lines overexpressing *TaGAPCp2* and *TaGAPCp3* after 25 days withholding water (Fig. 5a, b). Relative water content (RWC), a relevant tool for the measurement of drought tolerance, allows credible evaluation of the plant water status. The total chlorophyll content reflects the presence or absence of chlorosis. The contents of RWC and chlorophyll in transgenic lines were also higher than in WT after 15 days withholding water (Fig. 5c, d). Malondialdehyde (MDA), an important, indicator of membrane injury, was significantly higher in the WT than in transgenic lines after 15 days withholding water, suggesting that the transgenic plants suffered less membrane damage than WT (Fig. 5e). These results indicate that TaGAPCp2 and TaGAPCp3 all positively respond to drought stress.

**Fig. 5:** TaGAPCp2 and TaGAPCp3 responding to drought stress treatments in Arabidopsis. **a** Tolerance responses of the TaGAPCp2–overexpressing (OE-2) and TaGAPCp3–overexpressing (OE-3) lines to drought stress. Drought 25d: with holding water for 25d; R7d: resumption of water for 7 d after withholding water for 25d. **b** Survival rates of TaGAPCp2–overexpressing (OE-2) and TaGAPCp3–overexpressing (OE-3) transgenic lines, and WT plants on day 7 after resuming water following the withholding of water for 25d. At least 100 plants were counted and averaged for each line. **c** RWC of WT and transgenic lines after withholding water for 15d. **d** The chlorophyll contents of WT and transgenic lines after withholding water for 15 d. **e** The MDA content of WT and transgenic lines after withholding water for 15d. Error bars indicate ±SD (*n* = 3, from three technical replicates). Significant differences were assessed with one-sided paired t-tests (*, *P* < 0.05; **, *P* < 0.01). Three biological experiments were performed, which produced similar results

RETRACTED

### TaMYB interacts with *TaGAPCp2*P/*3*P

To gain further insight into the mechanism of transcriptional regulation, some Y1H reporter constructs were constructed to screen the wheat leaf cDNA library for gaining transcription factors. This screen indicated that TaMYB may bind to *TaGAPCp2*P*/3*P. As shown in Fig. 6b, cotransformation of the bait vector (TaGAPCp2P/3P in pAbAi) together with the individual prey vector of the identified interactor (TaMYB in pGADT7) into Y1H Gold yeast demonstrated interaction.

**Fig. 6:** *TaMYB* is transcriptional activator of *TaGAPCp2*P and *TaGAPCp3*P **a** Schematic diagram of the probes used for Electrophoretic mobility shift assays (EMSA) and fragments used for Yeast one-hybrid. **b** Yeast one-hybrid activity in TaGAPCp 2/3 promoter and TaMyb. **c** *TaMYB* bound MYB binding sites by EMSA.

To determine whether the TaMYB protein directly bound to *TaGAPCp2*P*/3*P in vitro, promoter fragments including the binding site at approximately 30 bp were used as probes for EMSA (Fig. 6a). The results showed that TaMYB could directly bind to the promoter fragments, and clearly demonstrated that transcription factor TaMYB can directly bind to *TaGAPCp2*P*/3*P and influence the transcription level (Fig. 6b).

### TaMYB interacts with a specific binding site to improve the transcription levels of *TaGAPCp2*P*/3*P under drought stress

To further validate the contribution of TaMYB to *TaGAPCp2/3*′ transcription levels under drought, a series of vectors with a 5′-deleted *TaGAPCp2*P*/3*P fragments and tested for their relative expression of Rluc/Fluc after drought stress (Fig. 7a, b). After 24 h of treatment with 20% PEG 8000, there were significant differences in the relative enzyme activity of Rluc driven by the serially 5′-deleted *TaGAPCp2*P*/3*P fragments. Figure 7c indicates that the fragments of *TaGAPCp2*P (− 1312~0) and Fig. 7c indicates that the fragments of *TaGAPCp3*P (− 2049~0) had some drought-related cis-elements.

**Fig. 7:** Screening of the *TaGAPCp2*P and *TaGAPCp3*P. **a**, **b** Schematic representations of the constructs containing a series of deletions of the T*aGAPCp2*P and *TaGAPCp3*P. **c**, **d** The relative expressions of Renilla luciferase in transiently transformed tobacco leaves. F1 to F7 represents tobacco leaves transformed with the dual luciferase reporter vectors driven by a series of deletions of the *TaGAPCp2*P (C) and *TaGAPCp3*P (D). The indicated values are the average of three independent experiments. The standard deviation (SD) is indicated at each point. Significant differences between treated and untreated (control) conditions were assessed with one-sided paired t-tests (*, *P* < 0.05; **, *P* < 0.01)

To further investigate which MYB binding site in the above fragments could be bound by TaMYB, we used the effector and reporter to instantaneously cotransform tobacco (Fig. 8a). We found that TaMYB interacted with the specific MYB binding sites of *TaGAPCp2*P (− 1197~ − 635) and *TaGAPCp3*P (− 1456~ − 1144 and − 718~ − 610) in plant cells (Fig. 8b, c). The Y1H system and EMSA demonstrated that the MYB binding sites in *TaGAPCp2*P (− 1135 and − 985) and *TaGAPCp3*P (− 1414 and − 665) were the TaMYB’ target cis-element (Fig. 9). These MYB binding sites connected with transcription activity were further assessed by deleting such site (Fig. 10a). The deletion of the MYB binding site in the promoter fragments all significantly restrained promoter’ activity responding to water stress (Fig. 10c, d). This confirmed that these MYB binding sites in *TaGAPCp2*P (− 1135 and − 985) and *TaGAPCp3*P (− 1414 and − 665) played vital roles in improving transcription levels under drought. The MYB binding sites in the *TaGAPCp2*P (− 1135 and − 985) and *TaGAPCp3*P (− 1414 and − 665) are all 5′-AACTAAA/C-3′ sequences and different from the other MBS. These results confirmed that the 5′-AACTAAA/C-3′ sequences are the TaMYB’ specific target cis-element (Additional file 4: Figure S4).

RETRACTED

**Fig. 8:** Identification of fragments bound by *TaMYB* in these promoters. **a** Schematic diagrams of the effector and reporter used for transient transactivation assays in tobacco. **b**, **c** Transactivation activity reflected by RLUC activity of RLUC/FLUC ratio, B for *TaGAPCp2*P; C for *TaGAPCp3*P. Asterisks indicate the significant difference between treatment and control (*P < 0.05,**P < 0.01 or ***P < 0.001)

**Fig. 9:** Identification of MYB-binding site bound by *TaMYB* in *TaGAPCp2*P and *TaGAPCp3*P. **a** Schematic diagram of the probes used for EMSA and fragments used for Yeast one-hybrid. **b** Yeast one-hybrid confirming the MBS activities. **c**, **d** *TaMYB* bound MBS by EMSA, B for *TaGAPCp2*P; C for *TaGAPCp3*P

**Fig. 10:** Verification of MBS bound by *TaMYB* in promoter. **a**, **b** Schematic representations of the vectors designed for MBS verification. **c**, **d** The relative expression of RLUC in transiently transformed tobacco leaves with the vectors indicated in **a**, **b**. Asterisks indicate the significant difference between treatment and control (*P < 0.05,**P < 0.01 or ***P < 0.001)

### The expression of *TaGAPCp2/3* is regulated by TaMYB in the ABA signaling pathway

Similar to *TaGAPCp2/3*, the transcription level of *TaMYB* was also enhanced in wheat responses to abiotic stresses (10 mM H_2_O_2_, 100 μM ABA and 20% PEG8000) (Fig. 11a). Expression of *TaMYB* was induced to the highest level (34.26-fold and 29.83-fold) at 8 h after PEG and ABA treatment. *TaMYB* expression increased 5.52-fold after 2 h of H_2_O_2_ treatment and reached the highest level (21.33-fold) after 4 h followed by a decrease (Fig. 11a). This indicates that both *TaGAPCp2/3* and *TaMYB* were likely involved in a stress-related signaling pathway. To investigate whether *TaMYB* was also involved in the ABA-induced upregulation of the expression of *TaGAPCp2/3*, wheat protoplasts transiently overexpressing *TaMYB* were used. In the wheat protoplasts overexpressing *TaMYB*, the relative expression of *TaGAPCp2/3* was significantly higher than that in the control group (Fig. 11b). Furthermore, the ABA-induced increase in the expression of TaGAPCp2/3 (the highest level of 13.36-fold and 12.16-fold) in the control protoplast was also enhanced by the *TaMYB* gene (the highest level of 23.98-fold and 18.42-fold) under ABA stress (Fig. 11b). These results indicate that the *TaMYB* gene is crucial for ABA-induced upregulation in the expression of *TaGAPCp2/3*.

**Fig. 11:** *TaMYB* gene regulate the expression of *TaGAPCp*2 and *TaGAPCp3* in wheat protoplast. **a** Expression patterns of *TaMYB* under abiotic stresse challenge of PEG, ABA and H_2_O_2_. **b** The transient overexpression of *TaMYB* promoted the ABA-induced expression of *TaGAPCp2* and *TaGAPCp3* in wheat protoplasts. The protoplasts were treated with 100 uM ABA, and the relative expression levels of *TaGAPCp2* and *TaGAPCp3* were analysed by RT-PCR. The indicated values are the average of three independent experiments. The standard deviation (SD) is indicated at each point. Significant differences between treated and untreated (control) conditions were assessed with one-sided paired t-tests (*, *P* < 0.05; **, *P* < 0.01)

## Discussion

Drought stress signals undergo transduction and other processes in plants, which eventually cause changes in transcription factor accumulation and activity [30–32]. The relevant transcription factor binds to a specific cis-acting element on the promoter of the gene and induces expression related tolerance to the drought stress [33–35]. In our previous work, it was discovered that *TaGAPCp2* and *TaGAPCp3* had different expression patterns under drought stress, although both genes had similar functions in drought tolerance in transgenic Arabidopsis. To further investigate these findings, we cloned and analyzed the promoters of *TaGAPCp2* and *TaGAPCp3* genes. Bioinformation analysis indicate differences in the cis-acting motifs in the promoters of these two candidate genes, suggestive of certain differences in their regulation.

RETRACTED

To study these two promoters in detail, *TaGAPCp2P* and *TaGAPCp3P* were subcloned into the pC0390-GUS vector and the pC0390-RUC vector and then transiently transformed into tobacco plants. GUS staining and the Rluc ratio indicated that the activity of the *TaGAPCp2* and *TaGAPCp3* promoters could be induced by PEG, ABA and H_2_O_2_ stress. At the same time, GUS staining and GUS enzyme activity of Arabidopsis plants transformed with *TaGAPCp2P:GUS* and *TaGAPCp3P:GUS* were analyzed to understand the expression patterns of different promoters under abiotic stresses. The activities of the *TaGAPCp2* and *TaGAPCp3* promoters were almost the same under normal conditions, and they both had stronger activity under drought stress (Fig. 4). This can be considered another line of evidence that supports the role of *GAPCp* in drought response [36]. For the crop, the seeds are the crucial product for human. Along with the development of plant genetic engineering, protecting the seeds from potential genetic contamination becomes important. In this work, we found that promoters of *TaGAPCp2* and *TaGAPCp3* had strong activity in almost every tissue except the seeds. This may be useful for application in the genetic engineering of crop.

Regulation of gene expression at the transcriptional level is primarily controlled by a promoter and its cis-acting regulatory elements [37, 38]. Yeast one-hybrid technology is a classical method for studying the interaction between DNA and protein, and allows the effective isolation and identification of proteins that bind to specific DNA sequence [39, 40]. The interaction protein *Ta*MYB of *TaGAPCp2P/3P* was obtained by yeast one-hybrid system and verified accurately by EMSA assays. Naturally, many MYB binding sites were found on the *TaGAPCp2/3*promoter. Several earlier reports have illustrated the important role of *Ta*MYB in drought resistance [41–43]. In wheat, TaGAMyb might participate in the heat stress response [44], TaMYB2A enhanced tolerance to abiotic stresses in transgenic Arabidopsis [45]. TaMYB73 involved in salinity tolerance via regulation of stress-responsive genes [42]. Similar to these reports, in wheat, the transcription level of *TaMYB* was also enhanced responses to abiotic stresses (Fig. 11a). Thus, the 5′ deleted mutants, and the Y1H and EMSA assays were used to determine the MYB binding sites that could be bound by *Ta*MYB and associated with drought. The TAACTA/G type of MYBR cis-elements was specifically recognized by Arabidopsis MYB96 and might also be specific for the wheat [46]. HvGAMyb bound to the oligonucleotides containing the 5′-TAACAAC-3′ and 5′-CAACTAAC-3′ sequences of the endosperm-specific genes promoter regions to regulate gene expression during endosperm development [47]. This work illustrated that the 5′-AACTAAA/C-3′ type MYB binding sites in TaGAPCp2P (− 1135 and − 985) and TaGAPCp3P (− 1414 and − 665) were specifically recognized by TaMYB, which was a member of the R2R3-MYB subfamily and related to AtMYB91(AT2G37630.1) [48] (Additional file 3: Figure S3, Additional file 4: Figure S4).

RETRACTED

## Conclusions

This study demonstrates that the transcription factor MYB can induce the expression of the *TaGAPCp2/3* gene by binding to the MYB binding site (5′-AACTAAA/C-3′) on its promoter, thereby enhancing the resistance of the plant under drought stress. These findings offer a better understanding of the role of the *TaGAPCp2/3* genes in response to drought and related abiotic stress in wheat, which could be candidates for improving crop water use efficiency and future biomass production.

## Methods

### Plant materials and treatments

Wheat (*Triticum aestivum* L.cv. Chinese Spring), tobacco (*Nicotiana tabacum*, cv.NC89) and *Arabidopsis thaliana* (Ecotype, Columbia) seeds were used in this research. The seeds were provided by the D209 laboratory of the College of Life Science. Seeds were surface-sterilized and then cultivated in a glasshouse at 16/8 h (light/dark, 22/20 °C).

To treat the wheat seedlings, 10-day-old wheat seedlings were transferred into Petri dishes containing 20% PEG8000, 10 mM H_2_O_2_ and 100 μM ABA solution for 24 h. Samples from treated (PEG8000, H_2_O_2_ and ABA at 0, 2, 4, 6, 8, 12 and 24 h) plants were frozen in liquid nitrogen and stored at − 80 °C for RNA isolation. Meanwhile, 10-day-old wheat seedlings grown under normal conditions were sampled as a control. All of the experiments were repeated at least three times.

For the abiotic treatment of infiltrated tobacco plants leaves (injected with the recombinant plasmids), the infiltrated tobacco plants were sprayed with 20% PEG8000 solution, 100 uM ABA and 10 mM H_2_O_2_. After 24 h of abiotic stress treatments, the treated leaf samples were stored at − 80 °C after being frozen in liquid nitrogen until Luciferase activity was assessed. All of the experiments were repeated at least three times.

RETRACTED

Wild-type and transgenic Arabidopsis lines overexpressing *TaGAPCp2* and *TaGAPCp3* were used for drought tolerance analysis. The seeds were sown on 1/2MS medium containing 30 μg/mL hygromycin for 1 week at 23 °C under a 16 h light/8 h dark cycle. Seedlings in similar at growth states were then transplanted into containers filled with soil and watered regularly for 2 weeks. Three-week-old plants were subjected to water withholding for 25 days. One hundred seedlings from each line or control were used to detect survival after 25 days of detained water. After 15 days of withholding water, fresh seedlings were harvested to measure the contents of Relative water content (RWC), chlorophyll and Malondialdehyde (MDA).

### RNA extraction and qRT-PCR analyses

Total RNA was extracted with TRIzol from the wheat seedlings and converted to cDNA using the PrimeScript™ RT reagent kit (TaKaRa, Japan). After treatment of wheat seedings with drought stress challenges (PEG 8000, ABA and H_2_O_2_), the expression of specific ESTs in the *TaGAPCp2* and *TaGAPCp3* gene families was determined through qRT-PCR, which was performed using SYBR®Premix Ex Taq™ (Tli RNaseH Plus) (TaKaRa, Japan) according to the manufacturer’s instructions on a Bio-Rad CFX96 system (Bio-Rad Laboratories, USA). The primers (TaGAPCp2/3*-*F and TaGAPCp2/3-R, Additional file 5: Table S1) used in qRT-PCR had high specificity as determined by agarose gel electrophoresis and were also confirmed by sequencing PCR products amplified by all primer pairs. The mean expression and standard deviation (SD) were calculated from the results of three independent experiments. Data analyses and quantitation were performed as previously described [49].

### Isolation and bioinformatics analysis of *TaGAPCp2*P*/3*P

The primers used for promoter cloning were designed based on the sequence of the Triticum cultivar (AOTI010005895.1) and *TaGAPCp2/3* genes. The upstream sequences of the *TaGAPCp2/3* genes were amplified by the primers named 2PF/R and 3PF/R (Additional file 5: Table S1), named *TaGAPCp2*P*/3*P. The PCR products were purified and cloned into a pEASY-T1 vector. Several clones of each reaction were sequenced and analyzed using the Plant CARE database (http://www.bioinformatics.psb.ugent.be/webtools/plantcare/html/) [29] and PLACE (http://www.dna.affrc.Go.jp/PLACE/).

### Transient activity analysis of the *TaGAPCp2*P*/3*P in tobacco

To detect the activity of *TaGAPCp2*P*/3*P, we constructed fusion expression vectors by using the pC0390-GUS vector and the pC0390-RUC vector as the main frame. *TaGAPCp2*P*/3*P were cloned into the vectors pC0390-GUS (located before the GUS reporter gene) and pC0390-RUC (located before the Rluc reporter gene) to generate recombinant plasmids. These fusion constructs were transferred into tobacco by agrobacterium-mediated transient assays. The CaMV35S promoter was used as a positive control.

RETRACTED

The GUS activity was measured with histochemical assays as described previously [50]. GUS activity was normalized to protein concentration and expressed as nmol 4-methylum-belliferone/min*mg protein. The GUS measurement was repeated at least three times. Transgenic plant leaves were histochemically assayed to determine GUS activity in accordance with the staining procedure described by Jefferson with minor modifications [51]. In brief, samples were incubated in GUS reaction buffer (50 mM Na_3_PO_4_, at pH 7.0, 2 mM X-gluc, 0.5 mM K_3_Fe[CN]_6_, 0.5 mM K_4_Fe[CN]_6_, 10 mM EDTA, and 0.1% Triton X-100) for 24 h at 37 °C. Stained tissues were incubated in 70% ethanol at 37 °C for 6 h to remove chlorophyll and then rinsed in 90% ethanol at 37 °C for 10 h. Finally, GUS histochemical staining was observed under a microscope. Firefly luciferase and renilla luciferase were assayed using the dual luciferase assay reagents (Promega, USA). Data were collected as the ratio of LUC/REN. All transient expression experiments were repeated three times. The data were analyzed using SPSS12.0 software.

### Generation and stress treatments of transgenic Arabidopsis

The full-length *TaGAPCp2*P*/3*P regions were amplified by PCR using specific primers (Ta1301–2/3F and Ta1301–2/3R). Then, the amplified products were cloned into the vector *pCAMBIA1301* and located before the GUS reporter gene. The resulting plasmids were separately used in transformation mediated by Agrobacterium (*Agrobacterium tumefaciens*) to obtain transgenic Arabidopsis lines. Transformed plants were cultured on 1/2 MS medium containing 30 mg/L of hygromycin and 0.8% agar at 22 °C for 2 weeks and then transferred to soil.

Homozygous T3 seeds of transgenic lines were used for the GUS activity analysis. Arabidopsis seeds were grown on 1/2 MS agar plates that were routinely kept in darkness for 3 days at 4 °C to break dormancy and then transferred to a tissue culture room at 22 °C. For abiotic stresses, 2-week-old seedlings were individually transferred to 1/2 MS agar plates containing 20% PEG 8000, 100 uM ABA and 10 mM H_2_O_2_ for 24 h. Samples from treated or control plants were frozen in liquid nitrogen and stored at − 80 °C until detecting the activity of GUS. All of the experiments were repeated at least three times.

### Yeast one-hybrid screening and electrophoretic mobility shift assays (EMSAs)

Fragments of the *TaGAPCp2*P*/3*P were cloned into plasmid pAbAi (TaKaRa, Japan) to screen the cDNA library, and screening of the cDNA library was performed according to the manufacturer’s instructions (Matchmaker One-Hybrid system; Clontech Laboratories Inc., Palo Alto, CA, USA) in the presence of 20 mM Aureobasidin A (AbA).

RETRACTED

A total of 100 ng of a 30 bp double stranded probe and 1 μg of purified *Ta*MYB were used in the EMSA reactions. After incubation at room temperature for 40 min, the samples were loaded onto a 6% native polyacrylamide gel. Then, the gel was poststained with Invitrogen™ SYBR™ Safe DNA Gel Stain and imaged with a Bio-Rad gel documentation system to detect DNA.

## Additional files

Additional file 1: **Figure S1** Nucleotide sequences of *TaGAPCp2* and *TaGAPCp3* promoters. (DOCX 658 kb)

Additional file 2: **Figure S2** Detection of transgenic plant. **a** PCR analysis of *TaGAPCp2*P transgenic Arabidopsis. **b** PCR analysis of *TaGAPCp3*P transgenic Arabidopsis. (DOCX 159 kb)

Additional file 3: **Figure S3** A phylogenetic tree of MYB TFs. A total of 169 sequences were analyzed including one sequences of wheat MYB TFs derived from cDNAs cloned in this work. (GenBank accessions shown in the figure). (PDF 136 kb)

Additional file 4: **Figure S4** Analysis of functional MYB cis-elements in the *TaGAPCp2* and *TaGAPCp3* promoters. (DOCX 246 kb)

Additional file 5: **Table S1** Primer and probe sequences used in this study. (DOCX 17 kb)

## Data Availability

The dataset supporting the conclusions of this article is included within the article and its additional files.

## Abbreviations

3-PGA: 3-phosphoglycerate
ABREs: ABA-responsive elements
DREs: Dehydration-responsive elements
EMSAs: Electrophoretic mobility shift assays
FLUC: Firefly luciferase
GAPCp: Glyceraldehyde-3-phosphate dehydrogenase in non-green plastids
GAPDH: Glyceraldehyde-3-phosphate dehydrogenase
GAREs: Gibberellin responsive elements
MYB: MYB transcription factor
qRT-PCR: Quantitative real time polymerase chain reaction
RLUC: Renilla luciferase
TPT: Triose phosphate transporter
Y1H: Yeast one-hybrid
